# Design of Intelligent Evaluation System for College Students' Mental Health Based on Big Data

**DOI:** 10.1155/2022/7119994

**Published:** 2022-07-13

**Authors:** Tao Hu, Xiaojun Zhang, Na Li

**Affiliations:** ^1^School of Medical Information Engineering, Gannan Medical University, Ganzhou 341000, China; ^2^First Affiliated Hospital of Gannan Medical University, Ganzhou 341000, China; ^3^Gannan Medical University, Ganzhou 341000, China

## Abstract

The mental health problems of college students have attracted the attention of all sectors of society. In order to keep college students in a good mental state and effectively analyze their mental health, an intelligent evaluation system of college students' mental health based on big data is designed. Based on big data technology, this article constructs an intelligent evaluation system for college students' mental health, which is divided into six layers, namely, application layer, decision layer, interface layer, analysis layer, data layer, and basic layer. Then, the mental health data of college students were collected based on C/S architecture. On the basis of extracting and integrating data characteristics, six evaluation indexes of personality, will, emotion, depression, fear, and psychosis were screened, and then, the intelligent evaluation was completed according to the weight of indexes. On the basis of the preliminary verification of the performance of the system in this article, according to the comparative experimental results, the mental health data acquisition time of the system is less, the accuracy of data feature extraction and the recall rate of evaluation results are higher.

## 1. Introduction

Mental health refers to the various aspects of psychology and activity process in a good or normal state. The ideal state of mental health is to maintain intact character, normal intelligence, correct cognition, appropriate emotion, reasonable will, positive attitude, appropriate behavior, and good adaptation [1, 2]. Mental health is influenced by both heredity and environment, especially the upbringing style of the family of origin in childhood. Mental health is prominent in social, production, and life to maintain good communication or cooperation with others, and can well deal with various situations in life. Individuals can adapt to the developing environment and have perfect personality characteristics. Their cognition, emotional response, and volitional behavior are in a positive state and can maintain normal regulation ability. In life practice, people can correctly understand themselves, consciously control themselves, and correctly treat external influences, so as to maintain psychological balance and coordination, and have the basic characteristics of mental health [3, 4].

Affected by the pressure of life, work, and study, psychological problems often baffle all kinds of people. Taking college students as an example, in the face of high intensity of academic pressure and inevitable employment pressure, psychological level often produces drastic changes, and mental health is greatly affected. With the increasingly fierce competition in modern society, the competition of physical strength and intelligence is far from satisfying the development of society, and the competition of psychological quality is the core competitiveness of this era. If the psychological quality is poor, it will seriously affect the study and life and even more seriously affect the future development and employment [5]. The mental health of college students is related to their own growth and the future development of the country, and more and more tragedies caused by mental health problems occur in the society, which not only affect their own life and future, but also cause serious harm to their families and others. Therefore, the mental health problems of college students have attracted the attention of all sectors of society. Early detection of whether college students have mental health problems is conducive to timely treatment or auxiliary prevention programs to help students develop healthily, and it is also of great social significance to promote the stable operation of schools [6].

Reference [7] designed a woA-improved random forest-based mental health assessment system for college students. The system divides college students' mental health into nine dimensions: psychosis, paranoia, terror, hostility, depression, anxiety, interpersonal sensitivity, compulsion, and somatization. Then, according to scl-90 total score, Chinese Conventional Model Evaluation Guide, and College Students' Mental Health Evaluation Standard, the mental health data are processed and evaluated discretely. Reference [8] designed an RFC college student mental health evaluation system based on the whale optimization algorithm. The system first collected RFC college students' mental health data, and then according to the current five common mental health problems of college students and the relevant evaluation criteria and data processing, the whale optimization algorithm was used to complete the mental health evaluation, which provided the decision basis for college students whether to carry out psychological counseling and treatment. Reference [9] designed a college student mental health assessment system based on VPMCD. Firstly, from the social environment, campus environment, family environment, and personal environment, the main factors that affect the mental health of contemporary college students are analyzed in detail, and then, the evaluation index system of mental health is established by using analytic hierarchy process, and the numerical calculation method of each level index is given. On this basis, a mental health assessment model based on VPMCD was established.

However, in practical application, it is found that the above traditional intelligent evaluation system of college students' mental health has some problems such as timeliness and accuracy. Therefore, this study designed an intelligent evaluation system for college students' mental health based on big data. The design ideas are as follows:

1. Build the overall system structure from the application layer, decision layer, interface layer, analysis layer, data layer, and base layer.
2. Build a data collection model of college students' mental health based on the C/S architecture.
3. Extracting and integrating the data characteristics of college students' mental health.
4. Select 6 evaluation indexes of personality, will, emotion, depression, fear, and psychosis.
5. Assign value to index weight, and then, complete intelligent evaluation according to index weight.

## 2. Design of Intelligent Evaluation System for College Students' Mental Health

Based on big data technology, this study constructs an intelligent evaluation system for college students' mental health. Big data refers to the huge amount of data involved, which cannot be retrieved, managed, processed, and sorted into more active information to help enterprises make business decisions in a reasonable time through mainstream software tools. “Big data” requires a new processing mode to have stronger decision-making power, insight and discovery power, and process optimization ability to adapt to a massive, high growth rate and diversified information assets. The strategic significance of big data technology lies not in mastering huge data information but in the professional processing of these meaningful data. In other words, if big data is compared to an industry, the key to the profitability of this industry lies in improving the “processing capacity” of data and realizing the “value-added” of data through “processing.” Technically, big data cannot be processed by a single computer and must adopt distributed architecture. Its feature is that distributed data mining for massive data must rely on the distributed processing, distributed database, cloud storage, and virtualization technology of cloud computing. The system is divided into six layers, namely, application layer, decision layer, interface layer, analysis layer, data layer, and basic layer. The overall structure of the system is shown in Figure 1.

### 2.1. Hierarchical System Design

According to the overall structure of the college students' mental health intelligent evaluation system constructed above, the hierarchical design is carried out.

#### 2.1.1. Based Layer

The basic layer of the system is the database software, dynamic environment, network environment, and hardware equipment necessary for the construction of the system and is also responsible for data collection, which is transferred to the data layer for storage.

#### 2.1.2. Data Layer

The system data layer mainly includes mental health assessment database, expert team database, and student information database, which provides data support for the analysis layer.

The data layer also includes two parts: student information management module and online consulting module. Among them, the student information management module includes student registration and login and other related operations. Online psychological counseling services can be provided for students only after they log in successfully. After entering the function interface, students can view and modify personal information and other related operations. When the student information is modified, the system will immediately notify online teachers and students to contact. The online counseling module is mainly responsible for providing psychological counseling services for students. The system of psychological counseling for students is free of charge, and the main purpose of psychological counseling is to help students better understand themselves, at the same time to solve the students' mental health problems. In special cases, psychology teachers can also turn off the SMS notification function.

#### 2.1.3. Analysis Layer

The main work of the system analysis layer consists of two parts. One part is the classification of evaluation reference cases summarized based on existing evaluation results and the classification of mental health evaluation materials [10–12]. The other part of the work is to use big data technology as the basis to extract students' personality, emotions, preferences, and other characteristics.

The analysis layer includes two parts: psychological test module and psychological test topic management module. Among them, the psychological test module is the core module of the system, but also the functional module that students mainly use, which mainly contains the emotion test and social test submodules. According to the data results generated by the module, the mental health problems of college students are divided into three levels: serious, general, and potential psychological problems or no psychological problems, which correspond to the three levels of screening of the mental health intelligent evaluation system. The psychological test topic management module mainly manages the psychological test topic of the student mental health intelligent evaluation system. Among them, it mainly includes the operation of adding and deleting evaluation topics. Among them, the classification of topic types is completed by teachers, and the operation of adding and deleting psychological test topics is completed by administrators.

#### 2.1.4. Policy Makers

After the analysis, the results were transmitted to the decision-making layer of the system, which evaluated the mental health of college students based on the evaluation rule base and iterative optimization rules.

At the decision-making level, scale test and social software data analysis are combined to conduct research, and the scale test results include test topic, test content, test time, user information, and other contents. Field settings of the evaluation scale are shown in Table 1.

#### 2.1.5. Interface Layer

The system interface layer has SMS interface and data exchange interface, which can be connected to the system for data exchange.

#### 2.1.6. Application Layer

The application layer of the system feeds back the mental health evaluation results to the application layer through the interface layer and provides the evaluation results to college students through the mobile terminal or PC terminal.

### 2.2. Intelligent Evaluation Process Design

#### 2.2.1. Mental Health Data Collection of College Students

This study constructs a data collection model for college students' mental health based on the C/S architecture, and its overall structure is shown in Figure 2.

The server side uses the basic attributes of the measurement points to realize the mapping between the data source measurement points and the target measurement points and provides the client with the required information related to the mental health data of college students. In order to facilitate management and search, the attributes of measurement points are generally stored in real-time database, and the client can only save the copy without manual revision [13–15]. If the monitoring point configuration changes, the server will immediately push the modification information to the client and get the updated local copy.

Client management includes configuration management and real-time situation management. Configuration management can achieve rapid client basic information fusion, and real-time situation management can test the current client binding information, obtain the specific value of data link traffic, evaluate the client operating mode and form, and monitor the network communication, and complete independent management. In the process of mental health data collection of college students, the server side uses the identification string to sort out the logical relationship between the measurement points and the client side [16–18].

The specific collection process is as follows:

Step 1: Configure preprocessing. Configuration preprocessing is the basis of mental health data collection of college students. Firstly, double calibration of data is carried out to remove the point data that is not available in the mental health data source, so as to prevent the inaccurate data collection caused by the difference between the server side and the data source of the measurement point category [19, 20]. In the preprocessing stage, select some attribute values to complete the mapping table reconstruction, which can enhance the search rate, reduce the packet length, and improve the transmission quality.
Step 2: Data transformation. After reading the current mental health data from the source database, three data transformations are performed according to the point configuration. Numerical quadratic transformation can deal with unit and reference value of metadata. The one-to-many transform can solve the problem of a single source measuring point responding to several target measuring points and maintain the completeness of data collection by using the transform process.
Step 3: Data transfer. The important function of the acquisition model is data transmission [21, 22]. In order to enhance the timeliness of data transmission, data transmission is processed from the following two perspectives in the system interface layer:
  - The network link shall use the long connection mode. Due to the long distance between the data source and the target server, long connection is used for data transmission in order to obtain a faster transmission rate. If the amount of transmitted data is not large, periodically transmit heartbeat packets to keep the link stable and reduce network transmission disconnection due to timeout policies of routers and firewalls.
  - Use of variable-length packets. According to the data packet header message, realize the data overall verification, subcontracting and analysis. The variable-length packet pattern is shown in Figure 3.
  - The introduction of data caching in the transmission sector. Based on the collection characteristics of college students' mental health data, the data cache is substituted in the transmission plate. If the network fails in a short period of time, the data will be cached to the memory, and the system does not contain any running cost [23, 24]. If the collection model fails for a long time, the data will be saved in a local file to maintain the authenticity of the later collection results.

Figure 4 shows the data cache architecture of college students' mental health. In order to maintain the safety of college students' mental health data, thread-safe queues were used to reduce the correlation between functional plates of the model and achieve the goal of high-quality data collection when multifunctional plates of the model interact.

#### 2.2.2. Feature Extraction and Fusion of College Students' Mental Health Data

The characteristics of college students' mental health mainly include behavioral characteristics, attribute characteristics, content characteristics, and social relationship characteristics, among which behavioral characteristics refer to the user's behavior on social network, including likes, comments, and online browsing traces. Attribute characteristics refer to the user's individual information, including name, age, gender, occupation, and hobbies. [25, 26]. Content features include users' chat content and posts on social software. Social relationship features refer to the interaction between users in the whole social network, which is manifested in the number of mutual attention and fans.

Firstly, the validity of the collected data information is inferred. If it is valid, the collected data information is converted into the data form directly processed by the system, which requires the introduction of the concept of time window to extract the mental health features of college students. The scale data and users' social network data are converted in batches, and different samples are divided. One sample corresponds to one window. The data in this time window are used to complete feature extraction, and the feature extraction results are classified and labeled. The time window selected here is 24 hours in order to obtain more comprehensive mental health data information of college students.

In order to further excavate the mental health state of college students and obtain more accurate psychological characteristics of users, the multifeature fusion analysis is carried out on the mental health data of college students. The mental health data obtained from multiple channels are analyzed as a whole to provide a basis for intelligent evaluation.

Neural network is an effective nonlinear data fusion method, which can transform input space into hidden space and analyze data more conveniently in hidden space. Therefore, neural network has strong data processing ability, and meets the requirements of large-scale data processing and is suitable for multifeature fusion analysis.

Assuming that the transformation function used by the hidden layer in the neural network is Gaussian function, the radial basis function output by the first element is

(1) $$\begin{array}{c} F\left(i\right)=\exp\;{\left(-\frac{\sum_{i=1}^{n}x_{i}-y_{i}}{2\partial^{2}}\right)}^{2}, \end{array}$$

where *x*_*i*_ represents the input quantity of mental health features of unit *i*, *y*_*i*_ represents the feature transformation quantity of unit *i* in the hidden layer, and *∂* represents the control parameter of unit *i*.

By inputting and extracting the characteristic data of college students' mental health and calculating the radial basis function according to the above formula, the multifeature fusion processing of college students' mental health data features can be realized.

#### 2.2.3. Determine Evaluation Indicators

Scl-9 mental health measurement form is the standard for the evaluation of indicators in this study. The selected evaluation indicators are personality *I*1, willpower *I*2, emotion *I*3, depression *I*4, fear *I*5, and psychosis *I*6, and the target layer is mental health evaluation. The psychological test data of college students in a certain university in recent three years were collected, and 90 samples were randomly selected as mathematical model samples according to the scl-90 scale integral method. The statistical results are shown in Table 2.

#### 2.2.4. Intelligent Evaluation of College Students' Mental Health

In this article, the mental health evaluation module in the decision-making layer of the system uses analytic hierarchy process to evaluate the mental health of college students. First, assign a value to the index weight and then complete the intelligent evaluation according to the index weight. The specific process is as follows:

Step 1: construct the judgment matrix model. Use 1–9 scaling and reciprocal measurement, and compare the importance of one indicator to another indicator pairwise, according to the comparison results to construct judgment matrix *J*.
Step 2: Use formula (2) to obtain the eigenroot solution of matrix *J*, and obtain the weight value of importance between the corresponding index of the same level and another index after normalization. Then, perform consistency test on the judgment matrix, and the process is as follows:
  (2) $$\begin{array}{c} \sigma J=\mu_{\max}\sigma^{-1}, \end{array}$$
*σ* and *μ*_max_ represent eigenvectors and maximum eigenvalues, respectively.
In the implementation of consistency test, the critical index value *C*_*I*_ of each matrix should be calculated first, and the random consistency index *R*_*I*_ should be searched at the same time, and the random consistency *C*_*R*_ can be obtained through calculation:
  (3) $$\begin{array}{c} C_{R}=\frac{C_{I}}{R_{I}}, \end{array}$$
where *C*_*I*_ and *R*_*I*_ represent the consistency index and consistency ratio, respectively. When the value of *C*_*R*_ is less than or equal to 0.1, it is proved that the hierarchical single-sort structure has a relatively suitable consistency. When *C*_*R*_ value is greater than 0.1, the index value of the matrix needs to be obtained again:
  (4) $$\begin{array}{c} \left\{\begin{array}{c} \mu_{\max}=\sum_{j=1}^{m}\frac{{\left(\sigma J\right)}_{j}}{\left(\sigma J_{j}\right)}\\ CI=\frac{R_{\max}-m}{m-1} \end{array}\right., \end{array}$$
where *m* represents the dimension of the matrix.
Step 3: use expert evaluation method to calculate index weight. Experts score the indicators based on rules relating to mental health status. The results can avoid the subjective opinions in the expert reference opinions and have rationality and objectivity.
Assuming that there are *k* experts, *k*_*I*_ represents the scoring value of experts for each indicator, then the weight calculation formula of mental health evaluation indicators is as follows:
  (5) $$\begin{array}{c} \omega_{I}=\sum_{1}^{k}\frac{k_{I}}{k}. \end{array}$$
Step 4: construct independent factor evaluation matrix. Let the fuzzy subset of factor *U*_*I*_ be *u*_*I*_, and obtain the membership degree of each evaluation index of mental health status through expert judgment method. When there are *κ* experts whose judgment grade of factor *U*_*I*_ is *L*_*I*_, the evaluation matrix expression formula is as follows:
  (6) $$\begin{array}{c} V=\frac{\kappa \times u_{I}\times L_{I}}{k}. \end{array}$$
Step 5: Use the linear weighted sum of objectives to construct intelligent evaluation, and the process is as follows:
  (7) $$\begin{array}{c} M=\sum_{I=1}^{6}\frac{V\times P_{I}\times \omega_{I}}{k}. \end{array}$$
where *P*_*I*_ represents the scoring value of item *I*. Input the extracted mental health feature data of college students, and calculate the target linear weighted sum according to the above formula, so as to realize multifeature fusion, further mine the mental health status of college students, obtain more accurate user psychological features, and conduct multifeature fusion analysis on the mental health data of college students. Analyze the mental health data obtained from multiple channels as a whole to provide basis for intelligent evaluation. The calculation process of target linear weighting sum is an effective nonlinear data fusion method, which can transform the input space into hidden layer space, and it is more convenient to analyze data in hidden layer space. Therefore, it has strong data processing ability, meets the needs of large-scale data processing, and is suitable for multifeature fusion analysis, so as to complete the design of College Students' mental health intelligent evaluation system.

## 3. Experiment and Result Analysis

In order to verify the practical application effect of the above designed intelligent evaluation system for college students' mental health based on big data, the source of mental health data of college students is the knowledge base of machine learning data set, which collects open datasets contributed by data scientists participating in machine learning projects; the following test process is designed.

### 3.1. Experimental Design

The simulation environment test system was built under MATLAB software. Experimental environmental parameters are shown in Table 3.

The experiment invited 50 students from the third grade of a university as the research object, including 25 boys and 25 girls. During the period of school, the experimental subjects generally have excellent academic performance and good comprehensive development.

First of all, preliminary validation is carried out to verify the quality of the system application indicators and the stability of the system. Then, the woA-improved random forest college student mental health evaluation system in reference [7] and RFC college student mental health evaluation system based on the whale optimization algorithm in reference [8] are compared. Comparative verification was carried out from the three perspectives of data acquisition time of college students' mental health, data feature extraction accuracy, and recall rate of the evaluation results.

Finally, the system is applied to test the mental health of 50 students and comprehensively analyze the mental health of college students from the perspectives of social factors, family factors, and personal factors.

### 3.2. Test Analysis

#### 3.2.1. Preliminary Verification

First, verify the quality of the system application index and the stability of the system. The system login interface is shown in Figure 5.

On the basis of assigning index weights, formula (4) is used to calculate the scores of each index, and the results are shown in Table 4.

As can be seen from Table 4, the calculation results of index scores are between 0 and 1. The score is divided into different grades: 0.9-1 is excellent, 0.8-0.9 is good, 0.7-0.8 is good, 0.6-0.7 is passing, and 0.6 is poor. It can be seen that all the indicators in the index layer have reached the good level, indicating that all the indicators are of the same importance to college students' mental health evaluation.

Then, the number of system running threads was used as an indicator to measure the stability of the system, and the system stability was tested. The results are shown in Figure 6.

Analysis diagram 6 shows that with the increase in the system running time, the system thread count showed a trend of rise at first and then remained stable, and 15 hours before the system running, the system number of threads increases slowly, but the increase is not obvious, and when the system running time exceeds 15 hours, the number of system running threads always stays within the range (20, 60). It can be seen that the number of threads is stable and the running state of the system is always stable.

#### 3.2.2. Comparison Verification

Firstly, the mental health data acquisition time of different systems was tested, and the results are shown in Figure 7.

According to the results shown in Figure 7, with the increase in the number of experiments, the mental health data acquisition time of different systems also changes. The acquisition time of system of reference [8] rises first and then decreases, and the global maximum value is 8.1 min. The acquisition time of system of reference [7] fluctuates frequently, and the global maximum value is 7.9 min. In contrast, the collection time of system of this article is less, which is always less than 6 minutes, indicating that the timeliness of system of this article is higher.

Then, the accuracy of data feature extraction is taken as the index to verify the reliability of different systems, and the results are shown in Figure 8.

By analyzing the results shown in Figure 8, it can be seen that when the number of experiments is 50, the data feature extraction accuracy of reference [7] system and reference [8] system reaches their maximum. When the number of experiments is 40, the accuracy of data feature extraction of this system reaches the global maximum, which can reach 0.95. It can be seen that the data feature extraction accuracy of this system is higher, which shows that the reliability of this system is higher.

Finally, the recall rate of evaluation results of different systems was tested, as shown in Figure 9.

By analyzing the results in Figure 9, it can be seen that with the increase in the number of experiments, the recall rate of evaluation results of different systems shows a downward trend. After more than 30 experiments, the recall rate of the evaluation results of the system in this article is gradually stable, while the two comparison systems do not show a stable trend of data, and the recall rate of the evaluation results of the system in this article is always higher than that of the two comparison systems, indicating that the method in this article is more effective.

#### 3.2.3. The Practical Application

Fifty students were divided into groups on average, and the mental health status of 50 students was tested by using the system of this article. The proportion of factors leading to mental health status of students in each group was tested from the perspectives of social factors, family factors, and personal factors, and the mental health status of college students was comprehensively analyzed, as shown in Figure 10.

As can be seen from Figure 10, among the test results of the mental health status of the 5 groups of students, the primary factors affecting their mental health status are social factors, followed by family factors and personal factors. Among the students in the third group, the family factors are lower than the personal factors, which is due to the difference of test subjects. In the five groups of assessment, social factors accounted for more than 70%, and family factors accounted for the highest proportion of about 32%; it can be seen that the social environment and small family environment are the main factors affecting students' mental health status, and compared with social and family factors, personal factors accounted for a relatively small.

To sum up, the designed intelligent evaluation system of college students' mental health based on big data has good performance, all indicators in the index layer reach a good level, and all indicators have the same importance to the evaluation of college students' mental health. In this article, the number of threads is stable when the system is running, and the running state of the system always remains stable. The acquisition time is less, which is always kept below 6 min, and the timeliness is higher. The data feature extraction of this system has higher accuracy and reliability. Social environment and family environment are the main factors affecting students' mental health. Compared with social factors and family factors, personal factors account for a relatively small proportion.

## 4. Conclusion

In order to provide effective data support for college students' mental health project, this study designed an intelligent evaluation system for college students' mental health based on big data.

Based on big data technology, the system of this article builds an intelligent evaluation system for college students' mental health on the basis of designing six layers: application layer, decision layer, interface layer, analysis layer, data layer, and basic layer. Then, based on the C/S framework, the mental health data of college students are collected and the data characteristics are extracted. Secondly, six evaluation indexes—personality, will, emotion, depression, fear, and psychosis—were screened, respectively, and then, the intelligence evaluation was completed according to the index weight.

In the experiment, the quality of the application index of the system is good and the stability of the system is high. After comparison and verification, it is found that the mental health data acquisition time of the system is less, the accuracy of data feature extraction and the recall rate of evaluation results are higher. Finally, a comprehensive analysis of the mental health of college students is made with the practical application of the system of this article.

## Figures and Tables

**Figure 1:** Overall structure diagram of intelligent evaluation system for college students' mental health.

**Figure 2:** Structure diagram of data collection model for college students' mental health.

**Figure 3:** Schematic diagram of mental health packet pattern of college students.

**Figure 4:** Data cache architecture diagram of college students' mental health.

**Figure 5:** System login interface.

**Figure 6:** System stability test results.

**Figure 7:** Comparison of mental health data collection time of different systems.

**Figure 8:** Statistical graph of data feature extraction accuracy of different systems.

**Figure 9:** Comparison diagram of recall rate of evaluation results of different systems.

**Figure 10:** Mental health assessment and analysis.

**Table 1:** Evaluate the field setting of the scale.

The serial number	The field name	The field type
1	Test topics	The integer
2	Content of the test	Character
3	Test time	The date type
4	The user information	The integer

**Table 2:** Scl-90 scale score.

Evaluation indicators	The serial number					The mean	The variance
	1	2	3	…	90		
*I*1	1.44	1.77	1.45	…	1.21	1.55	0.59
*I*2	1.41	1.70	1.86	…	3.35	1.87	0.70
*I*3	1.67	1.10	1.40	…	2.90	1.90	0.71
*I*4	1.65	1.12	1.42	…	2.19	1.86	0.72
*I*5	1.11	1.85	1.27	…	2.25	1.55	0.55
*I*6	1.44	1.90	1.63	…	2.45	1.74	0.66

**Table 3:** Experimental environmental parameters.

Parameter	The numerical
Runtime environment	Java 1.8
Server memory	16 GB
CPU	Intel Core i-2410 m
Programming language	Java
The hardware carrier	Fourth- and third-generation B raspberry pie

**Table 4:** The score of each index.

Evaluation indicators	Weight of indicators	Index scoring
*I*1	0.4841	0.9460
*I*2	0.1385	0.8643
*I*3	0.0457	0.7120
*I*4	0.0174	0.8325
*I*5	0.2600	0.7605
*I*6	0.1433	0.88326

## Data Availability

The raw data supporting the conclusions of this article can be obtained from the corresponding author upon request.
